The article "Clinical Effect of Virtual Reality Technology on Rehabilitation Training of Sports Injury" was retracted in 2023. Reasons: signs of a paper mill; suspected computer-generated content; unreliable results or conclusions; lack of ethics approval or compliance.

# Clinical Effect of Virtual Reality Technology on Rehabilitation Training of Sports Injury

**DOI:** 10.1155/2021/1361851

**Published:** 2021-10-11

**Authors:** Jing Chen

**Affiliations:** Yunnan University Dianchi College, Kunming 650228, Yunnan, China

## Abstract

In order to make most patients recover most of their limb functions after rehabilitation training, virtual reality technology is an emerging human-computer interaction technology, which uses the computer and the corresponding application software to build the virtual reality environment. Completing the training tasks in the virtual environment attracts the patients to conduct repeated training in the game and task-based training mode and gradually realizes the rehabilitation training goals. For the rehabilitation population with certain exercise ability, the kinematics of human upper limbs is mainly analyzed, and the virtual reality system based on HTC VIVE is developed. The feasibility and work efficiency of the upper limb rehabilitation training system were verified by experiments. Adult volunteers who are healthy and need rehabilitation training to participate in the experiment were recruited, and experimental data were recorded. The virtual reality upper limb rehabilitation system was a questionnaire. By extracting the motion data, the system application effect is analyzed and evaluated by the simulation diagram. Follow-up results of rehabilitation training showed that the average score of healthy subjects was more than 4 points and 3.8 points per question. Therefore, it is feasible to perform upper limb rehabilitation training using the HTC VIVE virtual reality rehabilitation system.

## 1. Introduction

Hemiplegia patients participating in practical rehabilitation training can gradually recover most of the functions of the affected limb. Effective rehabilitation training requires patients to participate in repeated rehabilitation training purposefully and actively for a long time. Stroke rehabilitation takes a long time and requires high training intensity, which requires a long period in the recovery process after stroke [1]. However, traditional rehabilitation training is challenging to provide high-level rehabilitation training services for hemiplegia patients due to the differences in the technical level of therapists. Repeating the same tedious exercise over a long period can reduce the patient's motivation to participate in rehabilitation training [2]. However, according to the theory of neurological rehabilitation, patients' autonomous participation in training is conducive to the recovery of neurological function in the process of rehabilitation training. Therefore, the movements of rehabilitation training need to be carefully designed, and patients need to actively participate in rehabilitation training for a long time and complete rehabilitation training tasks.

The article "Clinical Effect of Virtual Reality Technology on Rehabilitation Training of Sports Injury" was retracted in 2023. Reasons: signs of a paper mill; suspected computer-generated content; unreliable results or conclusions; lack of ethics approval or compliance.

Virtual reality technology creates a virtual environment through highly configured computers, related equipment, and specialized application software and lets people immerse themselves in the virtual environment. Virtual reality technology allows users to achieve a high level of presence [3]. By applying virtual reality technology to rehabilitation training, a task-oriented rehabilitation training system can be established. In this system, patients can conduct simulated training in virtual daily scenes, increasing their initiative to participate in training. Therefore, with the development of computer hardware and technology, virtual reality technology has been introduced into the upper limb rehabilitation training system and studied at home and abroad.

The repetition of a single action in rehabilitation training determines the dullness and unclear goal of rehabilitation training. Through the high-speed computing power of the computer, virtual reality technology transmits computer-generated images to the observer to create an immersive feeling [4, 5]. Then, the observer interacts with the virtual reality scene through specific virtual reality equipment, and the sense of immersion is strengthened again. The introduction of virtual reality technology into rehabilitation training can enable patients to participate in rehabilitation training actively. Through game tasks, patients can complete rehabilitation training while completing the task [3, 6].

A task-oriented VR rehabilitation training system is designed and developed for the VR device HTC VIVE. When patients wear the device for rehabilitation exercise, it can interact with the virtual environment to improve the efficiency and interest of rehabilitation training.

Virtual reality (VR) technology is a potential tool for cognitive process assessment and rehabilitation. The application research of virtual reality technology in rehabilitation training is developing continuously. Hwang et al. explored the effects of robot-assisted (RA) virtual reality (VR) intervention on motor function (MF) and neurological function (NF) in patients with stroke (CS) [7]. Montoya et al. outlined the application of immersive virtual reality-assisted rehabilitation technology in gait rehabilitation of stroke patients and compared it with traditional rehabilitation methods [8]. Hwang et al. discussed the effects of virtual reality-based upper limb rehabilitation training on upper limb function, muscle activity, daily living activities, and quality of life of stroke patients [7]. Abbas et al. discussed the effect of graded motor rehabilitation and cognitive function training supported by virtual reality (VR) technology on the efficacy of patients with CHF complicated with cognitive impairment [9]. Soufi Ahmadi et al. discussed the application of virtual reality technology in balance function rehabilitation training teaching, providing references and suggestions for using virtual reality technology in balance function rehabilitation training teaching [10]. Farshad et al. evaluated the influence of virtual reality (VR) training on the daily participation of different types of patients through a meta-analysis [11]. Moon and Jeon evaluated the effects of physical and cognitive training based on virtual reality on executive function and dual-task gait of elderly MCI patients and compared physical and cognitive training based on virtual reality with traditional combined physical and cognitive training [12]. Boroumand et al. observed the effect of virtual reality technology for balance training and conventional balance training on balance function of stroke patients with hemiplegia and carried out rehabilitation nursing and rehabilitation training for all patients [13]. Gokeler et al. discussed the effects of virtual reality training (VRT) and isokinetic exercise training (IKT) on the clinical and hormone performance of patients with chronic LBP [14].

The article "Clinical Effect of Virtual Reality Technology on Rehabilitation Training of Sports Injury" was retracted in 2023. Reasons: signs of a paper mill; suspected computer-generated content; unreliable results or conclusions; lack of ethics approval or compliance.

HTC VIVE, virtual reality equipment, designed and developed a virtual reality rehabilitation training system. Human upper limb movement is analyzed, a virtual reality system based on HTC VIVE is designed and developed, and finally, experimental verification is performed. Through repeated rehabilitation training, the purpose of upper limb rehabilitation training is achieved.

## 2. Research Methods

### 2.1. System Architecture of Virtual Reality Devices

HTC VIVE equipment wore end-to-end displays (HMD), a hand-held controller, and a positioner. Rehabilitation training users wore a display and a hand-held controller to interact with virtual objects in the real world. The locator captured the hand-held controller's location and rotary information and passed the data to the computer. After rehabilitation training system software for processing, the image was displayed on the head-mounted display and returned to the user [15].

In the subject, according to the activity rules of human upper limbs and the characteristics of the HTC VIVE interaction mode, three representative movements of hand moving to the specified position points on the desktop, hand touching the position point above the shoulder, and holding a cup to drink water were extracted. These movements were very close to the movements in life. In the design of the scene, the virtual room was selected as the scene to enable the patients participating in rehabilitation training to carry out rehabilitation training in a “comfortable” virtual environment, thus easing the mood of the participants and improving their enthusiasm for rehabilitation training.

The article "Clinical Effect of Virtual Reality Technology on Rehabilitation Training of Sports Injury" was retracted in 2023. Reasons: signs of a paper mill; suspected computer-generated content; unreliable results or conclusions; lack of ethics approval or compliance.

While participating in the training, the rehabilitation training patients controlled their hands in the virtual world to conduct human-computer interaction. There are two main ways of human-computer interaction: touch and grab. As shown in the figure, when the manipulator grasps the water cup to complete the drinking action, it triggers the two actions of touching and grasping. First, touch the water cup to the front of the body from the starting position of the action, and then use the trigger button of the hand-held controller to control the hand to grasp the water cup in the virtual world. Then, send the water cup to the mouth to complete the drinking action [16, 17]. During the whole experiment, the virtual hand completes all human-computer interactions as an object in the virtual world. Therefore, during the action mapping, the position coordinates of the virtual hand should be obtained to judge whether the actions performed at that time meet the training requirements through its movement trajectory.

### 2.2. Virtual Reality Training Scene Design

In the virtual world, objects need to be represented by various shapes of models, such as mountains, water, people, and animals. These objects need to be represented by modeling. The common modeling method is through modeling software. The simple schematic model can use the basic shape of the virtual reality engine for modeling. The success of a virtual reality scene depends on whether the user experiencing the virtual reality scene is immersed in the scene and whether the scene brings a strong sense of immersion to the user. It focuses on the light and shadow effect of the scene, the simulation effect of the model, and the physical constraints of the objects in the scene. The rehabilitation training environment set by this project is the living room in the family, so modeling technology is required to be used for modeling [18]. Unreal Engine 4 is used for rendering realistic light and shadow effects, and physical characteristics such as collision and gravity are given to the objects in the scene.

### 2.3. Experimental Steps

1. Debug the HTC VIVE rehabilitation training system to a normal working state, including system start-up, HTC VIVE operation room setting, rehabilitation training application software system start-up, and debugging.
2. The subject is seated on the chair, and the experimental table is located in front of the subject.
3. Adjust the height and position of the chair according to the experimenter's height and dominant hand (the default use of the right hand). First of all, make sure that the subjects' upper limbs move within a comfortable range during the experiment. Secondly, in the adjustment process, the height of the shoulder joint can be adjusted to make the subjects' sitting posture and movement more comfortable, with making the movement posture more standardized.
4. The volunteers in the experiment hold the controller and place it at point A 25 cm in front of the body.
5. Complete training actions 1, 2, and 3 according to the subject's ability.

The article "Clinical Effect of Virtual Reality Technology on Rehabilitation Training of Sports Injury" was retracted in 2023. Reasons: signs of a paper mill; suspected computer-generated content; unreliable results or conclusions; lack of ethics approval or compliance.

## 3. Results' Analysis and Discussion

### 3.1. Movements and Trajectories of Upper Limb Rehabilitation Training

This experiment extracted three rehabilitation training movements, which involved the shoulder joint's internal and external rotation and the elbow joint's flexion and extension. The training program of movement 1 is the movement of the wrist from starting point A to points B, C, and D, as shown in Figure 1.  Figure 2 shows an exemplary track record of the action one measurement.

As shown in Figure 2, when the hand moves to the specified position points on the table, the hand first lifts from the starting point of the action and then moves to the target position point in a parabolic shape. When an obstacle is encountered in the moving process, a breakpoint appears in the motion trajectory.

The training program of action 2 is the movement of the wrist from starting point A to the ipsilateral shoulder and then from the ipsilateral shoulder to the target point of the opposite shoulder, as shown in Figure 3.  Figure 4 shows an exemplary track record measured by action 2.

As shown in Figure 4, when the hand touches the position point above the shoulder, the hand is mainly a vertical upward movement.

The training program of action 3 is to grasp the water cup in the virtual world with the wrist from starting point A to D and then deliver the water cup to the mouth, as shown in Figure 5.  Figure 6 shows an exemplary track record of the action three measurements.

As shown in Figure 6, when drinking from a hand-held cup, the hands mainly move vertically up and in front of the body. Sparse track points reflect the speed of the hands at that time (the sampling interval is 10 ms, and the speed is slow when the hands are lifted).

This topic introduces a rehabilitation training system in a virtual environment. Due to the accurate tracking of HTC VIVE, the experimental results show that it is feasible to introduce HTC VIVE into upper limb rehabilitation, which increases the interest in rehabilitation training, and is suitable for family rehabilitation with low difficulty and cost.

The article "Clinical Effect of Virtual Reality Technology on Rehabilitation Training of Sports Injury" was retracted in 2023. Reasons: signs of a paper mill; suspected computer-generated content; unreliable results or conclusions; lack of ethics approval or compliance.

Future work will focus on people with different exercise levels and design exercise programs with different exercise intensities. So far, each movement has only one intensity. By setting different intensity training, it is expected to meet the needs of different groups of people. In addition, a more convenient interaction model should be designed with the rehabilitation robot of the upper limb exoskeleton to facilitate rehabilitation training for patients of different degrees.

### 3.2. Follow-Up of Rehabilitation Training

In the experiment, each set of movements should be repeated many times, and the frequency and amplitude of the movement can be adjusted autonomously. And keep the torso and head as still as possible while the arms are moving. Each session lasted about four minutes, and after completing two tests, participants filled out a Likert scale. The posttest questionnaire has a maximum score of 5 (1 is the lowest and five is the highest). The questionnaire aims to collect information on the accuracy, fun, and ease of using the HTC VIVE VR rehabilitation system.  Table 1 shows some of the questions included in the questionnaire.

Six subsequent patients were enrolled in the test. The purpose of the test was to initially check the effectiveness of the HTC VIVE and VR systems. Similarly, patients wearing an HTC VIVE head-mounted display led to three sets of actions. After completing the test, the patients filled out a questionnaire.

In the questionnaire results, as shown in Figure 7, the average score of the healthy subjects for each question was 4 points or above, and three patients also scored 3.8 points or above for the tie of each question. Therefore, it is feasible to use the virtual reality rehabilitation system of HTC VIVE for upper limb rehabilitation training. The highest score was for fun, with both the fitness testers and the patients scoring 4.8 or higher. The most significant difference in scores is the system usability, with an average score of 4.7 for the health test subjects and 3.8 for the patients. The reason is that the handle is not easy for the patients to hold and operate, so the exoskeleton auxiliary device can be introduced to design a better interactive way to use it. In addition, when a healthy tester experimented, one of the items gave 2 points. The reason was that the buttons of the handle were not easy to operate during the experiment. Therefore, the personnel involved in the rehabilitation training need to be trained before the rehabilitation training.

The article "Clinical Effect of Virtual Reality Technology on Rehabilitation Training of Sports Injury" was retracted in 2023. Reasons: signs of a paper mill; suspected computer-generated content; unreliable results or conclusions; lack of ethics approval or compliance.

## 4. Conclusion

The experiment of the virtual reality upper limb rehabilitation training system proves the feasibility of this system in rehabilitation training. The upper limb rehabilitation training program based on HTC VIVE virtual reality was formulated. The movement coordination, motion accuracy, movement completion, and HTC VIVE equipment usability index were qualitatively analyzed when the system was used for rehabilitation training. Finally, a questionnaire survey was carried out for the system. The analysis results further confirmed the system's feasibility, and some problems that should be paid attention to in clinical use were also found. To sum up, the virtual reality upper limb rehabilitation training system studied in this study is feasible, can increase the interest in upper limb rehabilitation training, and provide feedback and evaluation for rehabilitation training.

## Figures and Tables

**Figure 1:** Schematic diagram of training action 1: (a)wrist on table B, (b) wrist on table C, and (c) wrist on table D.

**Figure 2:** Motion track of the upper extremity in action 1.

**Figure 3:** Schematic diagram of training movement 2: (a) the wrist touches the target point on the same shoulder; (b) the wrist touches the target point on the other shoulder.

**Figure 4:** Motion track of the upper extremity in action 2.

**Figure 5:** Schematic diagram of training action 3: (a) the wrist reaches point D and grasps the cup; (b) the wrist delivers the cup to the mouth.

**Figure 6:** Movement track of the upper extremity in action 3.

**Figure 7:** Table of questionnaire evaluation data.

**Table 1:** HTC VIVE rehabilitation system evaluation questionnaire.

Serial number	The problem	Score
1	Is the enjoyment of using the equipment significantly improved compared to the rehabilitation training alone?	5
2	Is the virtual reality experience in a head-mounted display (HMD) realistic?	3
3	Does the action in virtual reality match the action in the real world?	4
4	Are you satisfied with the mission design?	3
5	After the task is completed, do these movements achieve the training effect?	5
6	Is HTC VIVE easy to use for upper limb rehabilitation training?	4

## Data Availability

The data used to support the findings of this study are available upon request to the author.
